The article "How does spectator presence affect football? Home advantage remains in European top-class football matches played without spectators during the COVID-19 pandemic" was published in 2021. Journal: PLoS One.

# How does spectator presence affect football? Home advantage remains in European top-class football matches played without spectators during the COVID-19 pandemic

**DOI:** 10.1371/journal.pone.0248590

**Published:** 2021-03-31

**Authors:** Fabian Wunderlich, Matthias Weigelt, Robert Rein, Daniel Memmert

**Affiliations:** 1 German Sports University Cologne, Cologne, Germany; 2 University of Paderborn, Paderborn, Germany; Queen Mary University of London, UNITED KINGDOM

## Abstract

The present paper investigates factors contributing to the home advantage, by using the exceptional opportunity to study professional football matches played in the absence of spectators due to the COVID-19 pandemic in 2020. More than 40,000 matches before and during the pandemic, including more than 1,000 professional matches without spectators across the main European football leagues, have been analyzed. Results support the notion of a crowd-induced referee bias as the increased sanctioning of away teams disappears in the absence of spectators with regard to fouls (p < .001), yellow cards (p < .001), and red cards (p < .05). Moreover, the match dominance of home teams decreases significantly as indicated by shots (p < .001) and shots on target (p < .01). In terms of the home advantage itself, surprisingly, only a non-significant decrease is found. While the present paper supports prior research with regard to a crowd-induced referee bias, spectators thus do not seem to be the main driving factor of the home advantage. Results from amateur football, being naturally played in absence of a crowd, provide further evidence that the home advantage is predominantly caused by factors not directly or indirectly attributable to a noteworthy number of spectators.

## Introduction

The COVID-19 pandemic in 2020 provides for the unprecedented chance to investigate the home advantage, as one of the most studied and best documented phenomena in sports [1, 2], in a natural experiment with matches taking place in the complete absence of spectators. This phenomenon (i.e. home advantage) is particularly evident in team sports (e.g. football [2, 3], basketball [4], ice hockey [5], American football [6], baseball [7]), but has also been reported to affect subjectively rated individual sports, such as gymnastics or figure skating [8]. However, the extent of the actual advantage for the home team can (clearly) differ between sports disciplines [1, 2] or individual regions or countries, where games are played [2, 9]. A good overview of the studies on the home advantage in various sports provide the meta-analysis of Jamieson [10] and the comprehensive review on the home advantage over time by Pollard and Pollard [2]. Researchers have tried to identify factors that can explain this phenomenon, and the most commonly discussed factors are briefly presented below. With regard to the previous literature [1, 11–13], these are crowd support, referee biases, psychological effects of expectations, travel fatigue, familiarity, territoriality, specific rules, and tactical behaviour.

A direct influence of spectators (crowd support) is discussed as a possible factor supporting the home advantage [5, 14], which is in line with the perception of the players [15] and the spectators themselves [16]. However, studies on the influence of absolute spectator numbers [4], stadium occupancy [5], or noise levels [17] have shown that spectators do not directly (or only to a very limited extent) take effect on the home advantage. Evidence for crowd-induced referee biases have been found in experimental studies [18] and real-world data [19–22], however, not all referee biases (although existent) actually contribute to the home advantage [23]. Psychological effects of expectation are based on the idea that players, coaches, fans, referees, and media are well aware of the phenomenon of home advantage and different expectations of the players at home and away matches [24] could have self-enforcing (increased home advantage) or self-locking (decreased home advantage) effects. Travel fatigue is assumed to be evoked by the longer and more stressful journey of the away team. The results of previous studies suggest that the absolute travel distance [25] and the number of time zones crossed [26], depending on the direction of travel [7], can contribute to the home advantage. Another potential influence on home advantage results from the (personal) familiarity with the sports facility [27, 28], possibly including constructional features, the nature of the playing field, and the unfamiliar conditions of the match preparation [27]. There is evidence that the home advantage is initially reduced if teams move to a new sports facility within the same city [27] and after the entire team has moved to a new city [28]. The factor territoriality refers to an increased hormonal reaction to defend own territory against attacks that can be observed in animal behavior. The idea to investigate territoriality as a possible factor contributing to the home advantage in sports is often attributed to Neave and Wolfson [13], who presented evidence for football players having higher testosterone levels prior to home matches, compared to away matches. The notion that rule factors contribute to the home advantage refers to certain rules that have the potential to directly or indirectly give a systematic advantage to the home team, such as batting last in baseball. However, there seems to be no rule in football distinguishing between home teams and away teams except for the choice of the shirt color, something that has been shown to be relevant in influencing the outcomes in combat sports [29], but unlikely to affect home advantage in football [30]. Adjusted tactical behavior could potentially be a consequence or a cause of home advantage. It is generally assumed that teams choose more offensive tactics, when playing at home compared to playing away [31], and there is evidence that this behavior is recommended by coaches [32].

Despite the overwhelming evidence of its existence and decades of research on this topic, the above-cited literature suggests that there is still no final consensus about the relative importance and interplay of different factors. It seems likely that more than one factor is responsible for the emergence of the home advantage and as it is almost impossible to experimentally manipulate real-world sports events, it is very difficult to disentangle the influence of different factors. Evidence can primarily be provided indirectly, for example by analyzing matches, teams or divisions with varying attendance [3, 33] and travel burden [25, 26] or by drawing conclusions from the characteristics of countries with a varying degree of home advantage [9, 34]. For a more direct analysis, it is promising to consider special circumstances, in which one or more factors can be virtually ruled out, such as same-stadium derbies [35], teams moving to a new sports facility or city [27, 28] or spectator exclusion due to hooligan violence [36]. These cases, however, are typically rare and thus studies have to rely on highly limited sample sizes. This has changed drastically due to the large number of matches played in complete absence of spectators as a consequence of the COVID-19 pandemic in 2020. We consider these matches as a natural experiment to investigate the contribution of spectators on the behavior of referees and players on the pitch as well as on the match results. To this end, differences between home and away teams with regard to disciplinary sanctions (fouls, yellow cards, red cards), match dominance (shots, shots on target), market expectation (betting odds), and the match results (goals, points) were analyzed. In addition, we included the results of amateur matches from low leagues, which represent another valuable source of matches without spectators.

In light of the above-mentioned literature on home advantage in general and referee biases in particular, we assume that the presence or absence of spectators influences disciplinary sanctions, match dominance, market expectations, and the home advantage itself, which is represented by the following hypotheses:

### 1 Disciplinary sanctions

The absence of spectators influences disciplinary sanctions (measured by fouls, yellow cards, and red cards) to the advantage of away teams.

### 2 Match dominance

The absence of spectators influences match dominance (measured by shots and shots on target) to the advantage of the away team.

### 3 Market expectation

The absence of spectators decreases the expected home advantage of the betting market (deduced from betting odds)

### 4 Home advantage

The absence of spectators decreases the home advantage (measured by goals and points)

## Methods

The influence of spectator presence on four different aspects of football matches is analyzed. First, spectators can be expected to influence the fouling behavior of players and the decision behavior of referees and thus might contribute to the home advantage. We make use of the number of fouls, as well as the number of yellow and red cards for each team in each match, as a reflection of fouling behavior and a possibly spectator-induced referee bias [19, 36]. Second, we investigate shots and shots on target, which can be considered to be measures of match dominance. Both have been shown to discriminate well between winning and losing teams in matches from World Cups, the Champions League, and domestic leagues [37–39]. Further, the number of shots [r(50538) = 0.29, CI = (0.28, 0.30), p<0.001] and the number of shots on target [r(50538) = 0.53, CI = (0.52, 0.54), p<0.001] are both significantly correlated to the number of goals scored by a team in the present dataset. Considering these additional match statistics has two advantages: The relatively higher number of occurrences in professional football matches (24.68 shots per match and 9.18 shots on target per match compared to only 2.64 goals per match in our database) leads to a decreased influence of randomness and thus, to more stable results. Moreover, these data enable further insights on the influence of game location on in-game processes. Third, we investigate the market expectation about the impact of spectator absence on the home advantage that is reflected in the sports betting market. Betting odds have been proven to be an excellent predictor of football matches [40–42] and (from a conceptual standpoint) should reflect all publicly available information, including the expectations of bookmakers and gamblers on the home advantage. Betting odds for the match outcomes (home win, draw, away win) were transferred to a forecasted probability for the respective outcome (for details on the calculation, we refer to Wunderlich and Memmert [43]). From these probabilities, the expected number of points gained from each team in each match was calculated. The advantage of expected points is that they are less susceptible to the inherent randomness in match outcomes, compared to goals and points. The disadvantage is that–although having a relatively high degree of efficiency–betting markets are not considered to be completely free from inefficiencies [44, 45]. Fourth and most importantly, we investigate the effects of spectator absence on the home advantage itself. Courneya und Carron [1] define (absolute) home advantage to be present if home teams win more than 50% of the matches. Common measures for the (relative) home advantage are based on the number of home and away wins when excluding draws [10, 46], on the number of points won at home and away [2, 9], or on the number of goals scored at home and away [19, 26]. Winner-based measures like the number of points are intuitive and widely used. At the same time, they do not come without limitations, as factors not related to the home advantage can have influence on the number of points gained at home and away. The competitive balance in a league is one such factor [9, 47], as the presence of very dominant or very weak teams can decrease the home advantage in terms of points. Other factors, like the overall number of goals scored in a league or different point systems, such as the three-point-rule, can have an influence on the number of draws [48] and thus have an effect on the total number of points. In light of the advantages and disadvantages stated above, the present paper makes use of both the number of points and the number of goals as a measure of home advantage.

### Data

The dataset includes professional football matches played under normal circumstances (i.e., in the presence of spectators), professional matches that were played without spectators due to the COVID-19 pandemic in 2020, and amateur matches in which almost no spectators are present anyways. With regard to professional football, we considered those countries being ranked under the top ten in the UEFA country coefficients at the end of season 18/19 (obtained from https://www.uefa.com/memberassociations/uefarankings/country/#/yr/2019), only leagues that were covered by the data source and a maximum of the two highest divisions per country. We excluded countries where the season was terminated prematurely (France, Belgium), where spectators were partially admitted during the COVID-19 pandemic (Russia) or that had a competition format deviating from a classical round-robin system (Ukraine). This results in a dataset of matches from ten professional leagues, including Spain, England, Italy, Germany, Portugal, and Turkey during the seasons 2010/2011 to 2019/2020. The dataset is split to matches being played under normal circumstances (N = 36,882) and matches played without spectators due to the COVID-19 pandemic (N = 1,006). The data exclude 32 matches that were not played due to an association decision or missing data. Moreover, we excluded data, where an inconsistent definition of shots and shots on goal was used (Premier League and Premiership in seasons 10/11–12/13 and Serie A in seasons 18/19–19/20). For each match, information on goals, points, betting odds for home win, draw, and away win (N = 37,888 matches), shots, shots on target (N = 21,714 matches) as well as fouls, yellow cards, and red cards (N = 25,270 matches) for home and away teams were collected from http://www.football-data.co.uk. Only matches in the usual round-robin competition format have been included, whereas knockout matches to decide on promotion or relegation at the end of the season were not considered.

The dataset with regard to amateur football consist of matches from the German division called Kreisliga A, which is a very low division clearly representing leisure sports. It includes all matches of season 2019/2020 that were played until the early termination of the leagues due to COVID-19 in March 2020. Data for the number of points gained on match level, as well as the total sum of home goals and away goals from all 39 Kreisliga-A-leagues being part of the State Football Association of Westphalia (Fußball- und Leichtathletik-Verband Westfalen) were collected from http://www.fussball.de covering a total of 5,624 matches (compare Table 1 for further details).

**Table 1:** Information on the data set.

Professional football			
Country	League	Number of matches with spectators	Number of matches without spectators
Spain	LaLiga	3,689	111
	LaLiga2	4,477	122
England	Premier League	3,708	92
	Championship	5,411	108
Italy	Serie A	3,667	130
	Serie B	4,300	107
Germany	Bundesliga	2,977	83
	2. Bundesliga	2,979	81
Portugal	Primeira Liga	2,703	90
Turkey	Super Lig	2,971	82
Total	-	36,882	1,006
Amateur football			
Country	League	Number of matches with spectators	Number of matches without spectators
Germany	Kreisliga A	-	5,624

### Statistical analysis

A careful statistical design is needed to make sure that differences between matches with and without spectators are entirely attributable to the spectator absence and not affected by further factors. For this reason, linear mixed regressions models were fitted to investigate the influence of spectators on the eight measures of disciplinary sanctions, match dominance, market expectation, and home advantage using two different time horizons and controlling for possible effects of seasons or leagues. Although the analysis is not focused on differences between leagues, it is important to control for such differences across the 10 different leagues by including *League* as a random effect. Controlling for seasonal effects is more complicated as the home advantage might both be subject to long-term developments [2] and shifts between seasons. Shifts between seasons might be caused by the new composition of teams, possibly affecting travel burden and familiarity; or rule changes, including major issues, such as the introduction of the video assistant referees [49] possibly affecting referee bias. To prevent such changes from confounding the results, the first variant of the regression models is only based on data from the season 2019/20, i.e., excluding any data of matches from earlier seasons. The advantage of this approach is that possible shifts between the seasons can be ruled out as a confounding factor. The second variant of regression models makes use of the full dataset including prior seasons, while controlling for long-time effects by including *Season* as a fixed effect. The advantage of the second approach is the significantly increased sample size of matches with spectators. For each of the eight measures, we used the difference between home teams and away teams as dependent variable. *Spectator* is coded as a dummy variable being 1 if spectators are present, *Season* is coded as -9 to 0 for seasons 10/11 to 19/20. The advantage of this data specification is that the constant of each model refers to the model estimation for season 19/20 in matches without spectators. A significant constant therefore suggest that differences still exist currently and even in absence of spectators. The linear model also enables us to directly estimate percental changes that are evoked over time across seasons and by spectator absence (see Tables 2 and 3).

**Table 2:** Influence of spectators on football matches based on data from season 2019/20.

Dependent variable	Goals	Points	Expected Points	Shots	Shots on Target	Fouls	Yellow Cards	Red Cards
**Number of matches**	3,752	3,752	3,752	3,372	3,372	3,752	3,752	3,752
**Constant**	0.2256*** (0.0545)	0.3248*** (0.0838)	0.2836*** (0.0289)	1.0422*** (0.2497)	0.3767** (0.1147)	0.2613 (0.1821)	0.1511** (0.0562)	0.0020 (0.0145)
**Spectator**	0.0482 (0.0637)	0.0633 (0.0935)	0.1495*** (0.0318)	1.3412*** (0.2902)	0.4146** (0.1333)	-0.7426*** (0.1979)	-0.4788*** (0.0657)	-0.0340* (0.0170)
**Estimated differences by the model**								
**With spectators**	0.2738	0.3881	0.4331	2.3834	0.7913	-0.4813	-0.3277	-0.0320
**Without spectator**	0.2256	0.3248	0.2836	1.0422	0.3767	0.2613	0.1511	0.0020
**Reduction by spectators**	17.6%	16.3%	34.5%	56.3%	52.4%	154,3%	146.1%	106,3%

The table reports the results for a linear mixed regression model including Spectator as fixed effect and controlling for League as random effect.

* p < 0.05,

** p < 0.01,

*** p < 0.001

**Table 3:** Influence of spectators and season on football matches based on seasons 2010/11–2019/20.

Dependent variable	Goals	Points	Expected Points	Shots	Shots on Target	Fouls	Yellow Cards	Red Cards
**Number of matches**	37,888	37,888	37,888	21,714	21,714	25,270	25,270	25,270
**Constant**	0.2241*** (0.0553)	0.3219*** (0.0817)	0.2804*** (0.0298)	1.029*** (0.2639)	0.3729** (0.1222)	0.2510 (0.2018)	0.1510** (0.0552)	0.0021 (0.0142)
**Spectator**	0.1079 (0.0564)	0.1519 (0.0833)	0.1399*** (0.0278)	1.399*** (0.2729)	0.4577*** (0.1264)	-0.5890*** (0.1774)	-0.4470*** (0.0571)	-0.0334* (0.0149)
**Season**	-0.0045 (0.0032)	-0.0066 (0.0047)	-0.0062*** (0.0016)	-0.0552* (0.0219)	-0.0306** (0.0101)	-0.0094 (0.0131)	0.0036 (0.0040)	-0.0000 (0.0010)
**Estimated differences by the model**								
**With spectators (10/11)**	0.3724	0.5330	0.4764	2.8915	1.106	-0.2536	-0.2640	-0.0334
**With spectators (19/20)**	0.3320	0.4738	0.4203	2.4280	0.8306	-0.3380	-0.2960	-0.0313
**Reduction by seasons**	10.9%	11.1%	11.8%	16.0%	24.9%	-33.3%	-12.1%	-2.5%
**Without spectators (19/20)**	0.2241	0.3219	0.2804	1.029	0.3729	0.2510	0.1510	0.0021
**Reduction by spectators**	32.5%	32.1%	33.3%	57.6%	55.1%	174.3%	151.0%	106.6%

The table reports the results for a linear mixed regression model including Spectator and Season as fixed effects and controlling for League as random effect.

* p < 0.05,

** p < 0.01,

*** p < 0.001.

The above-specified models will help to answer the question whether home advantage exists at all if spectators are excluded. If this is the case, other factors must account for at least some of the advantage that home teams have in football matches and these might also be present in amateur football. To clarify whether there is a difference between professional and amateur matches in the absence of spectators, an additional model was fitted. The model uses the differences in points for all professional and amateur matches in season 19/20 (N = 9,376) as dependent variable and includes the two dummy variables *Spectator* and *Professional*. No additional model for goals was fitted as our database does not include the goal difference on a match level for amateur football. Instead, the ratio of total home and away goals for professional and amateur matches was compared using a χ2-test.

## Results

Fig 1 illustrates differences between home and away teams for the eight variables across ten seasons and splitting the last season into matches with and without spectators. Driven by spectator absence, it seems that the existing differences are eliminated (if not reversed) for fouls, yellow cards and red cards and clearly decreased for shots, shots on target, and expected points. For goals and points, however, results do not appear unambiguous. Fig 1 also reveals that even before the COVID-19 pandemic some variables show notable fluctuations across seasons or appear to be subject to slightly decreasing long-term trends. A careful consideration of time effects across seasons is therefore essential. Moreover, caution is warranted as some of the variables do not cover all ten leagues for all seasons and the figure does not account for possible effects of different leagues.

**Fig 1:** Mean differences between home teams and away teams with regard to the eight measures and 10 seasons. Grey areas refer to 95% confidence intervals. Season 19/20 is split into matches with (“Yes”) and without (“No”) spectators. Numbers for goals, points, and expected points are based on 37,888 matches. Please note that the data for shots and shots on target (21,714 matches) as well as fouls, yellow cards, and red cards (25,270 matches) does not cover all leagues for all seasons.

Table 1 summarizes results for the regression models based solely on the season 2019/2020. The advantage of home teams under normal conditions (spectator presence) are reflected in more goals, points, expected points, shots, and shots on target, as well as less fouls, yellow cards, and red cards. The effects of spectator absence for all variables are in the expected direction, i.e., the differences are decreased or even reversed. The coefficients for *Spectator* show that these effects are significant for all variables, except for the measures of actual home advantage, that clearly fail to reach significance (p = .449 for goals; p = .498 for points). Moreover, the constants indicate that differences for home advantage, market expectation, and match dominance are still significant in absence of spectators, suggesting that the advantage of home teams is not fully attributable to spectator presence. For disciplinary sanctions, no significant differences are present in absence of spectators anymore, except for yellow cards that show a slight home disadvantage with home teams receiving more yellow cards. This is clear evidence that the referee bias completely disappears or is even slightly reversed in empty stadiums.

Results for the models including the full dataset are presented in Table 2. The overall picture for *Constant* and *Spectator* is the same as for the data-poorer model, however, goals (p = .056) and points (p = .068) are now very close to reach significance. Moreover, the model estimates the reduction of home advantage by spectators to be about one third, while it was only about one sixth in the data-poorer model. Effects of season confirm the observation that the home advantage, the market expectancy of home advantage, and the match dominance for home teams are generally subject to a decreasing tendency. The model estimates that the home advantage has been reduced by about 10% over the last ten seasons before the COVID-19 pandemic and omitting the variable *Season* from the model would thus lead to an overstatement on the effect of spectators on home advantage.

In summary, the present data is clear evidence that referee biases disappear or are even reversed in absence of spectators and Hypothesis 1 can be confirmed. Moreover, the match dominance of home teams measured as differences in shots and shots on target is reduced by half in the absence of spectators, lending evidence in favor of Hypothesis 2. Hypothesis 3 can also be confirmed, as the market expectation on home advantage in empty stadiums significantly reduces by one third. Some caution is needed with regard to Hypothesis 4, with the home advantage being reduced, but slightly failing to reach significance. Moreover, the estimation of the reduction depends on the time period considered. The crucial question seems to be whether the reduction in home advantage was caused by the spectator absence or already happened at the start of the 2019/20 season. Fig 2 illustrates the differences in points and expected points over time for each month during 10 seasons. Without the horizontal dashed line indicating the COVID-19 break, it would be impossible to notice the transition from matches with to without spectators in the data. This is due to both the high monthly fluctuation and the fact that the home advantage shows a decreasing pattern even before the interruption of leagues due to COVID-19. The expected points, however, show a relatively stable pattern and a clear drop at the exact point of the spectator exclusion. This graphical analysis once again shows that the data on match outcomes does not allow for far-reaching conclusions to be drawn about the home advantage. At the same time, the development of expected points is an indication that the reduction at the beginning of the season (at least from the markets’ point of view) was rather random than based on systematic reasons.

**Fig 2:** Monthly development of the difference between home and away teams with regard to points and expected points. The solid line refers to expected points, the dashed line refers to points and the grey area to 95% confidence intervals for points. Solid vertical lines refer to breaks between seasons and the dashed vertical line refers to the interruption of the leagues due to COVID-19. Months with less than 50 matches occuring at the start (end) of seasons were assigned to the next (previous) month. Matches played shortly before the interruption, but in absence of spectators, were assigned to the first month after the interruption.

Even if the absence of spectators reduces the home advantage, the present data is clear evidence that the home advantage does not fully disappear and thus, is not fully attributable to direct crowd support or spectator-induced referee bias. This leads to the question whether a comparable degree of home advantage can be found in amateur football matches as well. Results of the regression on points [Constant: 0.3569 (0.0354), p < .001; Professional: -0.0318 (0.0909), p = .514; Spectator: 0.0639 (0.0979), p = .726] revealed that a significant home advantage in Kreisliga A matches exists and that there is no significant difference in comparison to professional matches without spectators. The analysis of home and away goals (1,478 compared to 1,251 for professional matches; 13,985 compared to 11,575 for amateur matches) likewise revealed no significant difference (χ2 = 0.285, p = .594). The analysis of amateur data therefore suggests that the phenomenon of non-spectator-induced home advantage is not exclusive for professional football and that the degree of home advantage in amateur leagues is comparable to professional leagues.

## Discussion

Given the unprecedented chance provided by the COVID-19 pandemic in 2020 to investigate the home advantage in a natural experiment, the results provide strong evidence that the presence or absence of spectators does have a major influence on in-game processes with respect to disciplinary sanctions and match dominance. In matches under normal circumstances (i.e., with spectators) home teams receive less disciplinary sanctions and are able to create more offensive actions compared to away teams, both results being in line with prior literature [19, 36, 50]. The difference in disciplinary sanctions disappears or is even slightly reversed when the crowd is absent, which supports the idea that spectator presence is likely to be the only or predominant reason for biased referee behavior. Moreover, it is consistent with the result of an experimental study, suggesting that referees use crowd noise as a cue to evaluate the severity of fouls [18]. In the absence of spectators, home teams were still able to create more shots and shots on target compared to away teams, which suggests that the advantage of home teams can only partly be explained by the presence of spectators. The most important and at the same time most surprising result of the present study is that neither the disappearance of differences in personal sanctions, nor the decreasing dominance in shots or shots on target translates directly to the home advantage itself. Depending on the time horizon analyzed, the home advantage is non-significantly reduced by about one sixth or almost significantly reduced by one third in absence of spectators.

We can only speculate about the reasons why the differences in in-game processes do not have a stronger impact on the home advantage. A possible explanation with regard to the referee bias would be that yellow cards do have a minor impact on the final result of a game and red cards do not occur frequently enough to have a major impact on the home advantage. This line of reasoning is consistent with Riedl et al. [23], who showed that a referee bias with regard to injury time does not contribute at all to the home advantage at all. However, it is in conflict with the results of Anders and Rotthoff [51], who reported a negative influence of yellow and red cards on winning probability. A possible explanation of why the difference in shots and shots on target is not fully transferred to the home advantage is that shots can differ greatly in goal scoring expectancy, due to the position and characteristics of the shot [52]. Accordingly, in the presence of spectators, home teams might tend to take unpromising shots to unconsciously or consciously meet the expectations of their fans, who loudly yell for a shot, while not increasing the number of highly promising shots. This would result in a higher influence of spectators on the shots than on the results as observed in the data. Another conceivable explanation is that besides negative consequences, spectator absence could also induce positive effects for the home team, in line with the idea of choking under pressure [53, 54].

Between submission and revision of this paper, a highly related study [55] was published and claims a significant decrease of the home advantage in matches without spectators. While the study reports similar conclusions with regard to disciplinary sanctions and match dominance, the conclusions with regard to the home advantage differ. These differences can be mainly attributed to some weaknesses in the statistical analysis of the aforementioned paper. In particular, the authors included the number of goals and points for both the home and away team in a regression model, thus considering each match twice. Doing this includes observations to the analysis that are highly dependent on each other (e.g., three points at home always correspond to zero points away), which can artificially improve p-values. Moreover, due to this model specification, the inclusion of season and league effects does only control for the total number of goals and points, but not for differences between the teams, so that time changes in the home advantage over the last few years are not correctly reflected. This approach bears the risk of overstating both the magnitude and the significance of the effect of spectators on home advantage. Interestingly, this approach was only pursued for goals and points, but not for measures of match dominance or disciplinary sanctions.

Despite the above criticisms and our desire for cautious consideration, we do not want to deny a possible reduction of the home advantage caused by spectator absence. First, the mechanism that a decreasing referee bias and a decreasing match dominance will contribute to a reduction of the home advantage is highly plausible. Second, the betting odds indicate that the notable reduction of the home advantage prior to the COVID-19 break might be of random nature. Third, we also find a decreasing home advantage, yet insignificant and lower than stated by Scoppa [55]. Further data becoming available over the next months and years will help to determine the effect of spectators on the home advantage more precisely and with greater certainty. Follow-up studies should make use of these data and in particular focus on what happens once spectators will return to the stadiums.

Although the in-game processes are changing drastically, a significant degree of home advantage remains in empty stadiums. In the absence of the spectators’ direct crowd support, crowd-induced referee bias or any interplay of crowd presence with other factors, such as effects of spectators on familiarity, tactical behavior, or territoriality can be ruled out. Thus, the most important question is what drives the remaining home advantage? In particular as the data of the present study is based on the strongest European countries that are predominantly located in South-West Europe, where some circumstances, which seem to favor factors of the home advantage, are evidently not given. With regard to travel fatigue, no exceptional long distances between teams or travels, including different time zones, as common, for example, in North-American sports [7], are present. Likewise, countries with a recent violent history, which are assumed to possess a greater degree of territoriality [9], are not among the major leagues in Europe. Additionally, aspects increasing the role of familiarity, like large differences in pitch dimensions or quality of playing surface, as well as major differences in the altitude of stadiums [9], are rather limited in the big European leagues. In the introduction, rule factors have already been argued to be unlikely to contribute to the home advantage in the case of football. Although leagues from South-West European countries do not seem particularly exposed, a “normal” degree of travel fatigue, familiarity, and territoriality remain as plausible explanations for the occurrence of the home advantage. Further aspects that remain potential contributors are psychological effects of expectation and tactical behavior that could remain in matches without spectators, as coaches and players will still be aware of playing in a home or away match. An interesting argument in this regard is learned behavior that has been put forward by Staufenbiel, Riedl, and Strauss [46]. By investigating players in different youth leagues, the authors demonstrated that the home advantage increases with age, which could be explained by learning effects. Adapting this idea to the current data, it would be possible, that psychological expectation of increased home performance and corresponding tactical behavior persists (at least for some time), even if some actual causes of home advantage might not be present anymore.

By including matches from very low divisions of German football, we found evidence that a non-spectator-induced home advantage is not a phenomenon limited to professional sports, but can also be observed in amateur football. It has been shown that the home advantage in these amateur matches is comparable to the home advantage in professional matches without spectators. This is not a trivial result, as even in the full absence of spectators due to the COVID-19 pandemic some notable differences between regular amateur matches and professional matches can be identified. Accordingly, a similar degree of home advantage does not necessarily mean that the contribution of each factor may be equated. Travel fatigue, for example, is not a plausible factor in Kreisliga A, because of the regional character and the minimum distances between team venues. The familiarity of the home team with its own sports facility, on the other hand, can be assumed to be even more prominent in Kreisliga A than in professional football, as conditions vary considerably from one venue to the other, including varying pitch sizes and different types of surfaces, like grass, artificial turf or ash. Moreover, the influence of the aggressive behavior of individual spectators on referees, in particular through verbal threats of physical violence could cause an indirect referee bias even in absence of a large number of spectators. While amateur matches represent a nearly endless data pool of matches without spectators, solely points and goals, but no additional match statistics are available, making it difficult to shed more light on the effect of game location on in-game processes in amateur matches.

The probably unique number of professional matches played in the absence of spectators caused by the COVID-19 pandemic in 2020 resulted in a situation, where direct (crowd support) and indirect (induced referee bias) contributions of the fans on the match outcome can be fully neglected. However, the natural experiment in the present study is still subject to some limitations, that need to be considered.

Due to the fact that all games with spectators were played during non-pandemic times, while all games without spectators were played during the COVID-19 pandemic, it can be argued that this natural experiment is missing a real control group. This would be changed, if games at this level with spectators taking place during the pandemic were included. Unfortunately, this is not possible, as we are not aware of any league that is comparable in terms of playing level and data availability, but did not at least reduce the presence of spectators during the COVID-19 pandemic. Another possibility would be to analyze matches in absence of spectators that were played in non-pandemic times as has been done in the seminal paper of Pettersson-Lidbom and Priks [36] who analyzed empty stadiums in Italian leagues due to hooligan violence and safety concerns. While this approach solves the control group problem, it implies a very limited sample size for analysis and as matches without spectators were limited to stadiums with insufficient safety standards, the separation of control and treatment group cannot be considered completely random.

When drawing conclusions on the causes for home advantage, interactions between conceivable causes need to be considered [11], such as a possible influence of crowd presence on territoriality, familiarity, and psychological effects of expectations. Moreover, the quarantine and hygiene measures themselves could have caused a decreased familiarity for the home team. In light of the above discussion, only truly experimental designs would enable researchers to change a single factor in isolation and determine its contribution in an unambiguous way. However, such experimental designs would be far too costly and could never replace a real-world situation with all psychological effects present in a competition situation. This is one of the reasons why the difficult puzzle of the home advantage might never be fully resolved.

In the present study, disciplinary sanctions have been analyzed in an attempt to quantify referee biases. However, only data about the actual number of fouls called and cards awarded by the referees are available, while an objective evaluation of the situations is missing. If one team fouls more often and is penalized more often, this is not necessarily a reflection of referee bias, but of the fouling behavior itself. The data analyzed can thus be a reflection of both fouling behavior and referee bias and needs to be handled with some caution. In light of experimental evidence [18] and the fact that away teams are only sanctioned more often in presence of spectators, a referee bias seems to be the most plausible explanation.

In individual matches, the home advantage can be fully disguised by the strengths of the teams, which means that the clearly weaker team is still expected to be the outsider, even if playing at home. The home advantage in terms of goals and points thus can be confounded by the strengths of teams and researchers need to take care that datasets are not subject to biased team strengths (i.e. do not include a majority of strong home or away teams). If full seasons of data are used, this is considered to be unproblematic, as it implies that each match is played twice with either of the two teams enjoying the home advantage once. Due to the split of season into matches with and without spectators in the present study, this is not the case. However, due to the large number of timely connected matches considered and the fact that in the playing schedules a home match for a team is usually directly followed by an away match, the effect of the game schedule should be negligible. The present study does not control for a team-specific rating that captures for the inherent strength of each team at the time of each match (see [40, 43, 56] for discussion on this topic), which could be a valuable contribution of future work. Such ratings would help to demonstrate clearly whether the playing strengths are in fact completely equally distributed.

Two aspects that have not been tackled by the present study, but could be fruitful topics for further research, are the individual reactions of referees and teams to the spectator absence. it is conceivable that not all referees are equally affected by spectator presence. Unfortunately, the information on the match referee was not available at our data source for the large majority of matches and thus the present study did not account for differences in the individual reaction of referees. It could also be argued that individual teams react more strongly to the absence of spectators, possibly as these teams are used to a larger or louder home crowd. The present study did not account for the reaction of individual teams as prior research found no evidence for a team-specific home advantage [57] and the analysis of team-specific home advantage would require a separate methodological approach.

## Conclusions and practical implications

This paper sheds new light on the influence of spectators on referee biases and the home advantage by utilizing football matches in absence of spectators as a natural experiment. The present data is evidence that in absence of spectators the increased sanctioning of away teams disappears, the match dominance of home teams remains, but is decreased and the home advantage itself decreases, yet insignificantly.

Research on referee biases and the home advantage does not only help to understand these complex socio-psychological phenomena, but can also be relevant to referees aiming for objective decision making or team officials, coaches, and players trying to influence home advantage to their advantage.

In light of the present results, it actually seems to enhance success when teams consciously or unconsciously try to exploit biased referee behavior by putting as much social pressure as possible on referees through player behavior and spectator influence. The referees, who are expected to be as objective as possible in their decisions, should be specifically trained to meet these expectations even under high social pressure.

As the home advantage does not disappear in empty stadiums, there must be other contributing factors. Although the significance and interplay of such factors cannot be conclusively clarified, teams can at least try to strengthen the individual home advantage and reduce the individual away disadvantage through plausible measures. These could include attempts to increase familiarity in home matches, minimize travel exhaustion, stimulate territoriality or ensure that player expectation and tactical adjustments in away matches do not hinder success.
